# Study on the Application Effect of the Case Teaching Method Based on Primary Teaching Principle in Clinical Teaching of Radiology

**DOI:** 10.1155/2022/3448182

**Published:** 2022-08-17

**Authors:** Tong Gong, Yuting Wang, Hong Pu, Longlin Yin, Mi Zhou

**Affiliations:** Radiology, Sichuan Provincial People's Hospital, University of Electronic Science and Technology of China, Chengdu 610072, China

## Abstract

**Objective:**

A case-control study explored the application of case-based teaching methods in the clinical teaching of radiology.

**Materials and Methods:**

126 radiology interns of grade 2018 were selected by cluster sampling and randomly divided into the research group and the control group. The traditional teaching approach was used in the control group and the primary teaching principle was used in the research group. The teaching effects of the two groups were compared.

**Results:**

The interns' test scores, the research group's case summary multiple-choice questions, case-group multiple-choice questions, case analysis questions, theoretical total scores, and practical operation assessment scores were significantly higher than those of the control group, and the difference was statistically significant (*P* < 0.05). The total score of dimensions of the interns' critical thinking ability in the study group were significantly higher than those in the control group, and the difference was statistically significant (*P* < 0.05). The interns' perception of teachers, students' academic self-perception, students' perception of environment, students' social self-perception, and the total score of the DREEM scale in the study group were considerably greater than those in the control group, and the difference was statistically significant (*P* < 0.05). After teaching, the scores of systematic thinking ability and evidence-based thinking ability of the interns were significantly increased. The improvement in the study group was more significant than that in the control group, and the difference was statistically significant (*P* < 0.05). Following teaching, the scores of learning interest, self-management, plan implementation, and mutual cooperation of the interns in the two groups were significantly upregulated, and the difference was statistically significant (*P* < 0.05). Among them, the improvement of interns' abilities in the research group was significantly better than that in the control group, and the difference was statistically significant (*P* < 0.05). The scores of learning goal, learning process, learning effect, classroom environment construction, teaching strategy, and technology application in the research group were greater than those in the control group, and the difference was statistically significant (*P* < 0.05). The satisfaction rate of the study group was higher than that of the control group, and the difference was statistically significant (*P* < 0.05).

**Conclusion:**

The application of the case teaching method based on primary teaching principle in the radiology clinical teaching course is helpful to cultivate students' critical thinking ability and improve students' performance and classroom teaching effectiveness.

## 1. Introduction

The standardized training of radiology residents in China could be traced back to 1991. Through the standardized training in the department of radiology, the trainees can comprehensively grasp the imaging principle of common equipment in the department of radiology, the imaging manifestations of common diseases, and the differential diagnosis of some rare diseases [1]. How to better improve the clinical practice ability and post competence of radiology residents is an urgent clinical practice problem for imaging medicine teachers [2]. At present, the training mode in the clinical practice teaching of radiology is mainly based on the traditional teaching mode, but the teaching method centered on teachers, teaching materials, and topics can no longer meet the requirements of the hospital for medical students [3].

Typical case teaching method is a new teaching model in recent years. The typical case teaching method can not only encourage students to think independently and enhance their creative ability but also guide interns to combine theoretical knowledge with clinical practice. The classic case teaching method can guide students to actively think and summarize what they have learnt in time, making clinical practice teaching more vivid and concrete and achieve better teaching results [4, 5]. The primary teaching principle was first put forward by instructional design theorist Merrill in 2001. It is an important teaching principle summarized on the basis of studying various educational and teaching theories put forward by predecessors. It focuses on how to better facilitate learning and improve teaching effectiveness. The primary teaching principal advocates that under the purpose of “focusing on solving problems,” teaching should be carried out in a circle composed of activating old knowledge, demonstrating new knowledge, and applying new knowledge. It is a prescription teaching design principle to improve classroom teaching and attach importance to teaching effectiveness [6–8]. This principle completes the specific teaching tasks in a step-by-step situation of practical problems, which meets the requirements of learners' psychological development, so it is suitable for the practical course of internal medicine nursing which is closely connected with the clinic. Some scholars have tried to apply the primary teaching principles to the classroom teaching of surgery and geriatric nursing, which has displayed a good teaching effect [9–13]. The results of this study has indicated that the primary teaching principle is helpful to improve the interns' mastery of relevant knowledge and the ability to construct the knowledge system of radiology.

## 2. Materials and Methods

### 2.1. General Information

From October to December 2020, 126 interns in the Department of Radiology of grade 2018 were selected by the method of cluster sampling. All of them were enrolled in five-year clinical medicine major and randomly divided into two groups. There were 63 participants in the research group, including 52 boys and 11 girls. The age ranged from 20 to 23 (21.91 ± 0.93) years. The score of the first two academic years was (81.73 ± 0.22). There were 63 persons in the control group, including 50 boys and 13 girls. The age ranged from 19 to 23 (21.44 ± 1.36) years. The score of the first two academic years was (82.03 ± 0.45). There was no significant difference in age, sex, and performance between the two groups, so it was comparable.

Selective criteria are as follows: (1) all the participants had bachelor's degree regardless of gender; (2) the participants had no cognitive, language, and intellectual impairment, and had basic reading and writing ability; (3) they all participated voluntarily.

Exclusion criteria are as follows: (1) non-radiology interns; (2) those who could not cooperate to complete all the teaching tasks; (3) those who dropped out halfway or did not match well.

### 2.2. Methods

The interns in the control group carried out the traditional teaching mode and the teacher responsibility system for clinical teaching, which was mainly taught by the teacher, and the teaching content is completed in accordance with the practice syllabus. Theoretical knowledge and clinical skills in radiology were taught. Teaching activities are regularly scheduled on a weekly basis and the teaching program was regularly checked and feedback is given in a timely manner. Regular surveys were conducted to determine the satisfaction of the trainees with the teaching situation and to identify any problems in teaching. Finally, based on feedback from various sources, the teachers changed their teaching methods.

The interns in the research group adopt the case teaching method based on the primary teaching principle based on the control group. The specific methods are as follows: (1) Preparation before teaching. Two weeks before the formal start of the course, the leader of the research group conducted a two-hour collective training for the interns. The training content was related to the primary teaching principles, including concepts, basic elements, implementation steps, and operation methods of the e-teaching platform. Prior to the start of the class, the average grades of 63 interns from the previous two academic years were stratified into three tiers: upper, middle, and lower. Two to three interns were placed in each stratum, and seven to eight interns were placed in groups to ensure homogeneity between groups. Because of the practice syllabus developed by the radiology department, the representative frequently-occurring diseases and common diseases were selected. The cases were compiled by experienced medical teachers and experienced teachers and the real cases can be adapted. Case explanation can be combined with multimedia courseware and other forms, including clinical data, questions to be discussed, and reference answers. (2) Teaching methods would focus on the problem or complete task. One week before class, the teacher issued a case and a learning task list (composed of complete tasks and sub-tasks) [14]. The complete task was a general task designed by teachers on the basis of textbook and learning situation analysis, which was divided into easy to difficult subtasks in accordance with the principle of the task sequence, which required interns to complete the task. Subtask: (1) review and consolidate the theoretical knowledge of related diseases; (2) integrate the theoretical knowledge of various diseases and systems; (3) formulate targeted diagnosis and treatment plans. Before class, the group leader was responsible for assigning 8 contents, consisting of the case introduction, nursing evaluation, disease diagnosis, treatment goal, diagnosis and treatment measures, effect evaluation, health education, and disease-related knowledge to the group members, and then discussing and making PPT and mind map of case analysis ideas [15]. During this period, nursing students could log on to the case database of the e-teaching platform to refer to the uploaded literature, website links, and other related materials [16]. When analyzing the case before class, the group judged the type of disease according to the clinical symptoms, reviewed the main points of the knowledge of the disease again, and learned new knowledge. After the preclass discussion, each group of reporters made a centralized report and discussion to the teacher 2 days before class, and the teacher made suggestions for each group of reports and learned about the learning situation of nursing students in order to prepare for the lesson. (3) The content of new knowledge demonstrated by teachers should be consistent with the learning task list, combined with words, pictures, or videos to demonstrate the new knowledge in detail through analogy demonstration, picture imagination, intern debate competition, etc. [17]. After reviewing the old knowledge in class, 10 min was shown by 8 groups according to the mind map drawn by each group according to the diagnosis and treatment procedure in the form of slides to simulate the overall diagnosis and treatment process, which required that the disease diagnosis should be based on sufficient case basis. At the same time, when demonstrating new knowledge, we put forward relevant critical thinking problems and guide interns to use theoretical knowledge to solve problems step by step. (4) New knowledge was applied. As the interns gradually master knowledge, the teachers should gradually reduce guidance and finally provide interns with the opportunity to use new knowledge to solve variant problems [18]. The so-called variant problem was to change the problem situation around the teaching goal to make the interns follow suit [19]. (5) Convergence and integration. After first applying new knowledge to solve problems, interns needed further flexibility in selecting and applying new knowledge in real clinical cases in order to fully understand and integrate all aspects of knowledge [20]. The teachers needed to create opportunities for students to apply new knowledge flexibly. After classroom teaching, the students logged on to the e-teaching platform and learn similar cases of other causes in the case database. The cases came from real and complete clinical cases, which are closer to reality. The process of clinical diagnosis and treatment by learning the dynamic changes of the disease are practiced [21]. At the end of the self-study, the “discussion forum” of the e-learning platform course publishes the results of the case studies. The teacher guides students in speculation and communication.

### 2.3. Observation Index

#### 2.3.1. Course Assessment Results

After the end of the practical teaching course, the two groups of interns took part in the closed-paper examination of the same test paper. The research group compiled the question bank. The test paper types were 10 case summary multiple-choice questions (20 points), 5 case group multiple-choice questions (20 points), 2 case analysis questions (60 points) with a total score of 100 points. In the case analysis questions, candidates were required to carry out nursing assessment according to the disease profile (15 points), put forward disease diagnosis results and measures (30 points), and carried out health education (15 points). The papers were marked by teachers and there was a unified reference standard.

#### 2.3.2. Critical Thinking Ability

The Chinese version of critical thinking disposition critical thinking ability scale (CTDI CV) revised by Peng M.eici et al. [21] was used for evaluation. The scale included 7 dimensions, consisting of truth seeking, open mind, analytical ability, systematic ability, curiosity, self-confidence, and cognitive maturity. There were 10 items in each dimension with 70 items. Using the Likert 6-level scoring method, the scores were from 1 to 6 points from strongly disagree to strongly agree with the 70 to 420 points. The Cronbach's *α* coefficient of the scale was 0.90. It was uniformly distributed by teachers through the questionnaire star platform before the beginning of the course and after the end of the course. The effective recovery rate of the two questionnaires was 100%.

#### 2.3.3. Evaluation of Medical Education Environment

The DREEM scale was used for evaluation and five aspects were observed, including “students' perception of learning,” “students' perception of teachers,” “students' academic self-perception,” “students' perception of the environment,” and “students' social self-perception” [22]. To judge the problems were existing in the medical education environment, all items from disagree to strongly agree were expressed on a scale of 0 to 4 with a full score of 200. According to the total score of the scale, the educational environment was divided into 4 grades. The educational environment had serious problems (0–50 points); the educational environment had many problems (51–100 points); the educational environment was good (101–150 points); and the educational environment was very good (151∼200 points).

#### 2.3.4. Clinical Thinking Ability Score

The clinical thinking ability rating scale compiled by Roberts et al. was used to evaluate the thinking ability of the two groups of radiology interns before and after teaching, with a total of 24 items [23]. Through the Likert 5 grade scoring method, the score was positively correlated with the clinical thinking level. The content validity of the questionnaire was 0.89 and the reliability coefficient of Cronbach' *α* was 0.91.

#### 2.3.5. Autonomous Learning Ability

The autonomous learning scale was used to evaluate the self-learning ability of the two groups of interns before and after teaching [24]. The scale was divided into four dimensions, including learning interest, self-management, mutual cooperation, and plan implementation. The reliability and validity of the scale were 0.85 and 0.79, respectively.

#### 2.3.6. Evaluation of Teaching Effectiveness

The effective teaching evaluation form of the new curriculum edited by Sun Wenbo was used to evaluate the effectiveness of classroom teaching [25]. It was attended by other teachers who were not substituted by the project group. The dimensions of nursing students include three items, such as learning goal (10 points), learning process (30 points), and learning effect (20 points), which mainly evaluated the achievement of learning goals, nursing students' participation in activities and the level of intervention in problem solving. The teacher dimension included three items, consisting of classroom environment construction (10 points), teaching strategies (20 points), and technology application (10 points). The Cronbach's *α* coefficient of the scale was 0.89.

#### 2.3.7. Teaching Satisfaction

Self-developed teaching satisfaction questionnaire had a total of 100 points. More than 90 points were regarded as very satisfied, less than 60 points were regarded as dissatisfied, and others were regarded as satisfactory. Satisfaction = (very satisfied + satisfied)/100%.

### 2.4. Statistical Analysis

The research data were entered by two people. The *χ*2 test, *t*-test, and rank-sum test were carried out by SPSS25.0 statistical software. *P* < 0.05 indicated that the difference between the groups is statistically significant.

## 3. Results

### 3.1. The Examination Results between the Two Groups of Interns

First of all, we compared the test scores of the interns. The research group case summary multiple-choice questions, case group multiple-choice questions, case analysis questions, theoretical total scores, and practical operation assessment scores were significantly higher than those of the control group (*P* < 0.05, Table 1).

### 3.2. The Critical Thinking between the Two Groups of Interns

We compared the critical thinking of the two groups of interns. The total score of dimensions of the critical thinking ability of the interns in the study group were significantly higher than those in the control group (*P* < 0.05, Figure 1).

### 3.3. The Interns' DREEM Scale Scores between the Two Groups

We compared the scores of the two groups of interns on the DREEM scale. The total score of the DREEM scale were significantly higher than those in the control group, and the difference was statistically significant (*P* < 0.05). All results are shown in Table 2.

### 3.4. The Clinical Thinking Ability between the Two Groups of Interns

We compared the clinical thinking ability of the two groups of interns. Before teaching, there was no significant difference in the scores of systematic thinking ability and evidence-based thinking ability between the two groups (*P* > 0.05). After teaching, the scores of systematic thinking ability and evidence-based thinking ability of interns in the two groups increased significantly. Additionally, the improvement in the study group was more significant than that in the control group, and the difference was statistically significant (*P* < 0.05, Table 3).

### 3.5. The Scores of Learning Autonomy between the Two Groups of Interns

We compared the scores of learning autonomy between the two groups. Before teaching, there was no significant difference in all aspects of learning autonomy between the two groups (*P* > 0.05). After teaching, the scores of learning interest, self-management, plan implementation, and mutual cooperation of the two groups of interns were significantly higher than those before, and the difference was statistically significant (*P* < 0.05). Among them, the improvement of interns' abilities in all aspects in the study group was significantly better than that in the control group, and the difference was statistically significant (*P* < 0.05). The specific results are shown in Table 4.

### 3.6. The Classroom Teaching Effectiveness between the Two Groups

We compared the effectiveness of classroom teaching between the two groups. The research group scored significantly higher than the control group in the six items of learning objectives, learning process, learning effect, classroom environment creation, teaching strategies, and technology application (*P* < 0.05, Table 5).

### 3.7. The Teaching Satisfaction between Two Groups of Interns

We compared the teaching satisfaction of the two groups of interns. The study group was very satisfied in 34 cases, satisfied in 28 cases, and dissatisfied in 1 case, which the satisfaction rate was 98.41%. In the control group, 28 cases were very satisfied, 35 cases were satisfied, and 10 cases were dissatisfied. The excellent and good rate was 84.12%. The satisfaction rate of the study group was higher than that of the control group, and the difference was statistically significant (*P* < 0.05, Figure 2).

## 4. Discussion

As an important part of medical students' post-graduation education, resident clinical teaching is internationally recognized as a more scientific training method. The clinical teaching of residents is an important mean to train high-quality medical talents, which helps to improve the ability of clinicians in an all-round way. It is also a strategic measure to promote the steady improvement of a medical level in our country. Radiology department is one of the important departments of the hospital, which integrates examination, diagnosis, and treatment. Many types of diseases need to be diagnosed by radiology examination. Therefore, it is very important to train high-quality radiology staff. This study attempted to apply the primary teaching principle to the case-oriented practice course, and to explore the application effect of case teaching based on the primary teaching principle in the clinical practice course of radiology. The students' knowledge recall is improved and their ability to make comprehensive assessments and decisions is significantly improved. Firstly, during the activation of the old knowledge stage, the group creates a mind map before class. Students pay attention to uncovering the relevance of the systematic knowledge related to the case and form a structured knowledge. The simplified text and images can organize a large amount of relevant case information [26]. Therefore, students will deepen their memory and improve their mastery of knowledge on the basis of understanding knowledge. Secondly, in the stage of activating old knowledge and demonstrating new knowledge in class, the teachers explain the clinical knowledge not mentioned or less involved in textbooks. According to the case learning content reported by students, the new and old knowledge can be connected together to help students to further sort out and sum up case-related knowledge. In the stage of applying new knowledge, the students are able to apply new knowledge to practice for the first time and have a certain understanding of practical nursing procedures [27]. In the stage of integration, the students should learn similar cases based on the e-learning teaching platform. The construction of the students' knowledge system was made more systematic and structured through several practice sessions. The students' scores on case analysis questions requiring integrated understanding and decision-making have increased significantly. Finally, the interns in the research group realized more self-study and discussion of network resources based on the e-learning platform. The learning environment was easy, the degree of investment in learning was relatively high and the learning efficiency was high.

The intern DREEM scale was used to evaluate the students' comprehensive feelings of the medical education environment to find the weak links in the students' learning process. At the same time, it was possible to find the relevant contents of the hospital medical education environment that needed to be improved and provide strong evidence for improving the hospital clinical medical education environment. The scores of all dimensions of critical thinking ability of interns suggested that the primary teaching principle is helpful to the cultivation of critical thinking ability. The interns' perception of teachers, students' academic self-perception, students' perception of environment, students' social self-perception, and the total score of the DREEM scale were significantly increased. This means that the teaching environment of our college is better and the implementation of mind mapping teaching in the practice of medical imaging can improve students' clinical thinking ability in an all-round way. Critical thinking is a judgment process of logical reasoning, analysis, and evaluation of specific problems in some specific situations by scientific methods [28, 29]. Critical thinking is an abstract thinking skill, which emphasizes that students should practice and use it repeatedly in the process of solving problems [30]. Teacher-oriented case teaching is a one-way knowledge transfer. Case discussions are short and students are prone to confusion of knowledge and learning fatigue. However, case studies based on primary teaching principles can give students more opportunities to exercise their thinking. In the part of focusing on problems, students analyze and study various resources independently around learning task sheets. In addition, the group discussion draws mind maps to present the thinking process of case analysis to effectively exercise their ability to promote the construction of logical thinking and effectively improve the ability to find the truth and analyze. In the link of demonstrating new knowledge, the teachers give encouragement to the content of students' case reports, so that students can observe and associate in analogy. The internal relationship is found what they have learned to enhance students' self-confidence in autonomous learning achievements and improve their open-mindedness. In the application of new knowledge and integration, the students understand and integrate the learning content from various perspectives through variant case drills, which is conducive to the cultivation of systematic thinking.

In addition, this study has indicated that the primary teaching principle can effectively improve the effectiveness of classroom teaching. The increased effectiveness of teaching may be due to the teacher's ability to stay close to the students' knowledge base when developing completed tasks. The sequence of questions is reasonably broken down to form a list of learning tasks and students' learning objectives are more clearly defined. Group cooperative learning before class is more willing to express their own views and stimulate learning motivation. The teachers explain new knowledge in class, combining with pictures, animation, and texts to give timely and comprehensive guidance to students. A relaxed, warm, and positive learning environment can be created to improve the satisfaction of classroom teaching. There are some limitations in this study. First, the sample size of this study is not large and it is a single-center study, so bias is inevitable. In future research, we will carry out multi-center, large-sample prospective studies, or more valuable conclusions can be drawn.

In conclusion, the application of the case teaching method based on primary teaching principle in the radiology clinical teaching course is helpful to cultivate students' critical thinking ability and improve students' performance and classroom teaching effectiveness.

## Figures and Tables

**Figure 1:** The critical thinking between the two groups of interns.

**Figure 2:** The comparison of teaching satisfaction between the two groups of interns.

**Table 1:** The examination scores between the two groups of interns [$\bar{x}$ ± *s*, points].

Group	*N*	Multiple choice questions in case summary	Multiple choice questions of case group type	Case analysis questions	Total score of theory	Examination results of practical operation
R group	63	19.08 ± 1.21	18.19 ± 1.52	53.78 ± 2.73	53.76 ± 2.73	91.85 ± 1.84
C group	63	16.21 ± 1.65	17.24 ± 2.08	49.21 ± 3.55	49.25 ± 3.48	82.61 ± 2.11
*t* value		11.113	2.927	8.100	8.093	26.197
*P* value		<0.05	<0.05	<0.05	<0.05	<0.05

**Table 2:** The interns' DREEM scale scores between the two groups [$\bar{x}$ ± *s*].

Grouping	*N*	Students' perception of learning	Students' perception of teachers	Students' academic self-perception	Students' perception of the environment	Students' social self-perception	DREEM total score of the scale
Research group	63	33.22 ± 2.83	29.08 ± 2.41	23.07 ± 1.66	32.68 ± 3.62	19.89 ± 1.73	139.62 ± 6.44
Control group	63	31.58 ± 2.51	23.36 ± 2.01	16.37 ± 1.94	29.24 ± 3.01	15.44 ± 1.56	108.52 ± 5.92
*t* value		3.441	14.467	20.828	5.800	15.162	28.219
*P* value		<0.05	<0.05	<0.05	<0.05	<0.05	<0.05

**Table 3:** The clinical thinking ability of the two groups of interns ($\bar{x}$ ± *s*, points).

Grouping	*N*	Systematic thinking ability		Evidence-based thinking ability	
		Before teaching	After teaching	Before teaching	After teaching
Research group	63	30.36 ± 2.83	40.15 ± 1.48^b^	18.56 ± 3.87	26.38 ± 0.79^b^
Control group	63	29.83 ± 2.52	33.52 ± 1.84^a^	18.47 ± 3.31	20.49 ± 0.98^a^
*t* value		1.110	22.286	0.140	37.140
*P* value		>0.05	<0.05	>0.05	<0.05

*Note.* The comparison before and after teaching in the control group, a *P* < 0.05; The comparison of the research group before and after teaching, b *P* < 0.05.

**Table 4:** The learning autonomy scores between the two groups of interns before and after teaching (*x* ± *s*, points).

Grouping	*N*	Interest in learning		Self-management		Cooperate with each other		Plan implementation	
		Before teaching	After teaching	Before teaching	After teaching	Before teaching	After teaching	Before teaching	After teaching
Research group	63	18.33 ± 4.13	24.78 ± 3.37^b^	28.87 ± 4.36	35.84 ± 3.21^b^	13.19 ± 2.14	17.38 ± 3.63^b^	18.26 ± 2.51	23.81 ± 4.26^b^
Control group	63	19.12 ± 4.32	20.24 ± 3.76^a^	28.21 ± 4.51	31.27 ± 3.22^a^	13.26 ± 3.72	15.27 ± 3.81^a^	18.73 ± 2.84	20.26 ± 5.45^a^
*t* value		1.049	7.137	0.835	7.978	0.129	3.182	0.984	4.073
*P* value		>0.05	<0.05	>0.05	<0.05	>0.05	<0.05	>0.05	<0.05

*Note.* The comparison before and after teaching in the control group, a *P* < 0.05; the comparison of the research group before and after teaching, b *P* < 0.05.

**Table 5:** The classroom teaching effectiveness between the two groups (*x* ± *s*, points).

Grouping	*N*	Intern evaluation			Teacher evaluation		
		Learning goal	Learning process	Learning effect	Classroom environment construction	Teaching strategy	Application of technology
Research group	63	9.56 ± 0.23	28.11 ± 0.34	19.02 ± 0.56	9.38 ± 0.22	18.56 ± 0.72	9.12 ± 0.46
Control group	63	8.01 ± 0.14	20.07 ± 2.31	14.05 ± 1.21	7.26 ± 1.19	12.05 ± 2.33	7.05 ± 1.23
*t* value		46.691	27.331	29.587	13.905	21.188	12.511
*P* value		<0.05	<0.05	<0.05	<0.05	<0.05	<0.05

## Data Availability

The datasets used and analyzed during the current study are available from the corresponding author upon reasonable request.
